The article "Environmental Sustainability Impact of Environmental Protection Regulations on the BRICS Countries" was published in 2022. Journal: J Environ Public Health.

# Environmental Sustainability Impact of Environmental Protection Regulations on the BRICS Countries

**DOI:** 10.1155/2022/4626387

**Published:** 2022-08-28

**Authors:** Mingjun Liu

**Affiliations:** King's College London, London WC2R 2LS, UK

## Abstract

The BRICS countries are also known as the BRICS, which are composed of five economies: China, Russia, India, Brazil, and South Africa. Of course, environmental issues are also included, because with the economic development of the five countries, the price paid is the environment. In response to this problem, in order to adapt the environmental problems arising in their own development to economic development, the BRICS countries have formulated corresponding laws and regulations to respond to existing or possible environmental problems. The most important purpose of this series of environmental protection laws is to achieve relatively stable and sustainable development in the five countries. This requires these environmental protection laws to have a sustainable impact on the environmental development of the BRICS countries. In order to conduct research on the impact of sustainable environmental laws that have been enacted, this article will use the analysis method of analyzing the relationship between the environmental protection regulations and economic development of the BRICS countries, as well as the relationship between the environmental protection laws and environmental sustainability development of the BRICS countries, and the impact of environmental sustainability based on empirical analysis. It assesses the impact on the sustainability of the environment of the BRICS countries under the auspices of environmental laws. Through the empirical analysis experiment of economic and environmental protection effects, the results obtained show that the comprehensive scores of environmental protection in the BRICS countries in 2018–2020 have been improved except Russia's score. Among them, the improvement of China's score is the most obvious, and the improvement of the ranking has reached 24. The results of this assessment show that, with the support of the corresponding environmental laws, sustainable impacts have been produced in the environment of the BRICS countries.

## 1. Introduction

With the vigorous development of economy and technology in recent years, environmental issues have become issues that need to be considered in both developed and developing countries. This brings the concept of sustainable development to the development of the country. The sustainable development here mainly refers to not taking the environment in which human beings live as the price of development in the process of development and utilization of the environment and in the development of economy. And these environments are the environments that human beings will live in now and in the future. The importance of the environment to human beings has been clearly demonstrated in some developed countries this year, and it is also evident in some developing countries that regard the environment as the price of development. As five developing countries with obvious advantages in today's international environment, the BRICS countries have a relatively important influence on the development of the world economy. However, with the increasing number of environmental problems in the five countries, corresponding laws and regulations have been carried out on the protection of the environment. This measure enables environmental protection to have a legal basis, and to a certain extent, it can improve or even solve the environmental problems arising in development. In order to achieve sustainable development of the environmental protection efforts made by the five BRICS economies, this article will use certain methods to evaluate this phenomenon. It uses this to determine the role of environmental laws in the development of the BRICS countries.

The sustainable impact of the environment reflects the good relationship between human beings and the natural environment. The grasp of this relationship can well deal with environmental and economic risks, and many researchers have made relevant research. Khalid and Peng controlled energy consumption by assessing the sustainability impact of the environmental life cycle [1]. Brown was to obtain better economic benefits by studying the relationship between the sustainable impact of the environment and the business economy [2]. Ali et al. conducted an analysis of the sustainability impact of some of the world's resources by using environmental protection methods [3]. Bayar and Remeikiene reduced the emission of pollutants by improving the utilization rate of energy, which can make sustainable improvements to the environment [4]. Aziz et al. assessed environmental sustainability impacts using both qualitative and quantitative methods [5]. All of the above studies have been conducted with regard to the impact of environmental sustainability. These studies will demonstrate the various factors that have an impact on the environment. The measures involved are also various, and these methods can be classified as part of the implementation of environmental protection law. The main way is to control some energy consumption products. The use of these modalities allows for a partial demonstration of the reasons for having a sustainable impact on the environment. However, the use of these methods lacks an assessment of the impact on the environment after the implementation of the environmental protection law. In order to solve this problem, this article will use the method of empirical analysis to conduct qualitative and quantitative research on environmental problems.

With regard to the research on the continuous impact of environmental protection law on the environment, the method of empirical analysis is used to conduct research. The use of this method allows for a more objective presentation of the impact of environmental sustainability. And many scholars have discussed it. Wilson et al. conducted a structural analysis of environmental sustainability impacts by using an empirical approach [6]. Santos et al. quantitatively monitored changes in environmental sustainability impacts by using meteorological data obtained in the environment [7]. Dalavi et al. estimated the sustainability impacts of water resource occurrences in the environment by using empirical methods [8]. Vishi and Bhagat conducted an empirical analysis model of rainfall in the environment by using empirical analysis [9]. Flumignan et al. conducted an empirical analysis of meteorology in the environment by using sensors [10]. In the mentioned series of studies, the methods of empirical analysis are related to the impact of environmental sustainability. This makes this method more important in the evaluation of the sustainable impact of the environment under the action of environmental protection law. The role of the empirical analysis method in the study of the environmental sustainability impact is to analyze and process the environmental sustainability impact in the BRICS countries by means of statistical measurement. Using the empirical analysis to analyze the impact of environmental sustainability under environmental law can better clarify the relationship between environmental law and environmental change.

The status of the BRICS countries in the world is constantly improving with the economic development of each country in this group. The vigorous development of the economy in the five countries has made environmental problems increasingly prominent. Long before the establishment of this combination, the emergence of various environmental problems has led to the introduction of corresponding environmental protection laws in the BRICS countries. Environmental issues have become more and more important in recent years, and many concepts of green and sustainable development have also been proposed in the international community. However, the effect of the laws promulgated by the BRICS countries is largely based on qualitative concepts. In order to achieve sustainable development of the environment, it is not to slow down the economic development, but to use the environment as a sustainable resource while ensuring economic development. It is not about trading the environment for economic development. On the basis of using the empirical analysis method, through the empirical analysis experiment of pollutants, it is obtained that the laws of Brazil and Russia's investment in the environment are consistent. Brazil's investment is 21.71 billion yuan. After the investment of Russia is 42.38 billion yuan, it is a stable investment and the use of energy by the BRICS countries continues to increase in the use of energy in the world. By 2020, the use of industrial energy by the BRICS countries will reach 41.17%. These results show that environmental laws have a significant effect on environmental sustainability. That is to say, under the implementation of their respective environmental protection laws, the environment of the five BRICS countries has achieved sustainable green development to some extent. The innovation of this article is that it studies the impact of environmental laws on environmental sustainability. It also uses a certain method to explore the relationship between the two.

## 2. BRICS Environmental Sustainability Impact

### 2.1. Relationship between Environmental Protection Regulations and Economic Development

The BRICS countries are playing an increasingly important role in the international development environment, which also makes the cooperation between the five countries in the economic field closer and closer. Of course, the rapid economic development has brought great changes in people's lives and various aspects to the five BRICS countries, but with the economic development, there is also serious environmental pollution [11]. Until now, serious natural disasters have occurred. It has made the BRICS countries in developing emerging markets realize the importance of environmental protection to the country. The corresponding five countries have already promulgated corresponding laws and regulations, in order to achieve a better balance between the seemingly intractable environmental and economic development. Therefore, it is necessary to adopt a new mode of economic development and environmental protection based on the existing scientific and technological means. The new mode is shown in Figure 1.

Figure 1 shows a new model of environmental and economic development. The difference between this model and the traditional economic development model is that environmental regulations and the environment are placed at the beginning of the model. This also determines that this development model is not based on the pursuit of economic benefits, but rather on the environment. In order to better correlate the protection of the environment with the economic development of the BRICS countries, the laws and regulations in Figure 1 only regulate environmental protection. However, it is also necessary to carry out corresponding regulations for the industry that has the greatest impact on the environment in the BRICS countries, namely, the industrial industry [12]. Since the secondary industry is very important to a country, a country's industrial strength can determine its competitiveness in the international community to a certain extent. Therefore, a country's heavy industry is very important for its environmental protection and international competition, and it is also very important for the evaluation of the secondary industry. The evaluation system for the secondary industry is shown in Figure 2:

In the evaluation system in Figure 2 above, the characteristics involved in the production process of the entire secondary industry have been described as indicators. It also performs corresponding calculations for the key parts of the figure. From the above figure, we can also know that if the secondary industry undergoes major changes, it may affect the overall competitiveness of the country in the international community. The above indicators can be used as a reference indicator for the BRICS countries before and after the implementation of environmental protection. However, more environmental-related indicators need to be collected for environmental protection. These indicators are serious pollutants for the environment, but are indeed essential for industrial development. The corresponding indicators of environmental pollutants are shown in Figure 3:

The indicators involved in various industries shown in Figure 3 are highly dangerous pollutants for the environment, and the environmental damage caused by them is also relatively serious. When a country's industry develops rapidly, the short-term economy will be greatly improved, but it will be accompanied by a large amount of emissions of these pollutants. In dealing with environmental issues, the BRICS countries are not only unified in the evaluation system of the abovementioned pollutant indicators, but also reflected in the development of the environment, environmental technology, environmentally friendly energy, and related political decisions. In addition, the global greenhouse effect is becoming more and more serious. And the BRICS countries, which are developing and emerging countries, are now the major countries in greenhouse gas emissions. Various countries have made corresponding policies and analyzed the emission of pollutants.

### 2.2. Relationship between Environmental Protection Laws and Environmental Sustainability

The environment in which the environmental protection laws of the five BRICS countries are promulgated is the growing concern of the international community for environmental governance. At the same time, the importance of the BRICS countries on their national economic development has also reached a new height. Since the concept of globalization was put forward, the vast majority of countries in the world have made their own connections in development. The linkages between countries make developing countries an opportunity to pass on energy consumption in developed countries. Although it can bring economic growth, modern industry and some manufacturing industries that have obvious harm to the environment have also brought serious environmental problems to the environment of developing countries [13]. As the representatives of developing countries, in order to achieve sustainable development in terms of the environment, the BRICS countries need to combine the sustainable development of the environment of the five countries on the basis of the environmental protection laws issued by the five BRICS countries. Its sustainable development model incorporating the concept of environmental protection is shown in Figure 4.

The environmentally sustainable development model in Figure 4 provides a complete display of the environmental use model. The sustainable development of the environment here is to rationally arrange the environmental resources of the entire Earth at the two levels of time and space. The purpose of this is not to make too much sacrifice of environmental resources for short-term development. The coordination in Figure 4 is to place environmental protection on a longer span and a larger space, not just between the BRICS countries. Moreover, in the above model, the usability of the environment and the normativeness in use are effective measures for environmental protection. Sustainable environmental protection brings not only environmental benefits, but also better maintenance of stable economic development.

### 2.3. Method of Environmental Sustainability Impact

The principle of the empirical analysis method is to use some specific analysis methods in the practical analysis to process the data to a certain extent. The usage scenarios of this method are mostly processing economic data, and the corresponding analysis methods are also diverse [14]. What this article studies is the impact of sustainability under environmental issues, and the influencing factors and indicators involved can be roughly specified in terms of nature and quantity. The first is the calculation of the attribute indicators in the influencing factors. Now it is assumed that the national competitiveness of the BRICS countries is denoted by *K*, and the five countries' corresponding efforts to implement environmental protection in their own countries are denoted by *T*. When *K* appears alone, its corresponding probability is expressed as *P*_*kk*_. When environmental protection is simply analyzed from the perspective of protection, its corresponding probability is *P*_*tt*_. In the event of environmental protection, when neither the country's competitiveness nor the protection of the environment exist, the probability of occurrence is *P*_0_, and when both attributes are present, the probability of occurrence of the corresponding event is *P*_*KT*_. Because this article is about the impact on environmental sustainability, the abovementioned attribute indicators, that is, the relationship between the country's competitiveness and the strength of environmental protection, need to be related to a certain extent. First of all, it is necessary to determine the relationship between the competitiveness of the BRICS countries and environmental protection. The logarithmic analysis method is used here. The formula is as follows:

(1) $$\begin{array}{c} \ln\;P_{KT}=\ln\;P_{tt}+\ln\;P_{kk}+\ln\frac{P_{KT}}{P_{tt}P_{kk}}. \end{array}$$

The above formula expresses the logarithmic form of the two influencing factors specified in nature. However, these two factors must be two without interference before they are correlated. The establishment of this requirement needs to be based on the following formula:

(2) $$\begin{array}{c} \frac{\left(P_{kk}P_{tt}\right)}{\left(P_{KT}P_{TK}\right)}=1. \end{array}$$

The above formula mathematically correlates the competitiveness *K* of the attribute country with the environmental protection intensity *T* corresponding to the country. The ratio of 1 in formula (2) represents only the independence between the above factors, and the regulation of the correlation strength can be expressed as

(3) $$\begin{array}{c} \eta =\frac{\left(P_{kk}P_{tt}\right)}{\left(P_{KT}P_{TK}\right)}. \end{array}$$

The size of the *η* value in the above formula indicates whether there is a mathematically defined relationship between the country's competitiveness and the country's protection of the environment. It can be seen from the formula that when the value of *η* is more biased, it shows that there is a close relationship between the country's own competitiveness and the country's protection of the environment. The process of calculating the indicators of the nature category in the above content can also be extended to the influencing factors of other attribute categories, such as the relationship between the national environmental protection awareness of the BRICS and the strength of environmental protection. In addition to this, a mathematical definition of the influencing factors that can be monitored numerically is required. In Figures 2 and 3, an indicator system has been established for the pollution problems faced by the BRICS countries at the current stage of development [15]. As emerging economies of developing countries, the BRICS countries not only need to vigorously develop their own industries, but may also undertake the industrial production of some developed countries. The development of industries is very important for developing countries. There are three categories of indicators that are destructive to the environment, including sewage, gas, and solid pollutants. The indicators of the above three categories of pollutants are expressed as *H*_*ab*_. It represents the pollution index of pollutant *b* in year *a*. The weight of one type of pollutants in the whole can be expressed as

(4) $$\begin{array}{c} L_{ab}=\frac{H_{ab}}{\sum_{a=1}^{i}H_{ab}}. \end{array}$$

The above formula can calculate and express the respective weights of the three types of pollution. In order to better define the degree of confusion of a certain type of pollutant in the above pollution system, it can be expressed by the following formula:

(5) $$\begin{array}{c} \phi_{i}=\frac{1}{\ln\;20}\sum_{a=1}^{20}L_{ab}*\;\ln\;L_{ab}. \end{array}$$

The above calculation of the degree of confusion of pollutants in the pollutant system provides a good definition of the normative nature of pollutants. The above calculation process quantifies the pollutant indicators in industrial development in a very specific manner. Among them, formula (4) defines and calculates the weights of various pollutants in the industrial development of the BRICS countries. But in the end, the index of pollutants has to be calculated, and its formula is expressed as follows:

(6) $$\begin{array}{c} D_{r}=\sum_{b=1}^{p}k_{b}*L_{rb}. \end{array}$$

The calculation formula of the above pollution index has carried out a specific calculation of the specific detection values of environmental pollutants. The calculation form of the above expression formula can summarize the detection values under the corresponding weights of all pollutant indicators in a class of pollutants. In order to better correlate the environmental protection laws promulgated by the BRICS countries with the lasting impacts on the environment occurring in the five countries, the calculation methods of formula (1) and formula (3) are also required. It can better present the results of the impact from the quantification of indicator attributes and indicators.

### 2.4. Environmental Sustainability Impact Experiments and Results

The experiment in this article compares the impact of BRICS environmental protection law enforcement and environmental sustainability between quantitative indicators of pollutant reduction over a longer period of time and the gross domestic product of the national economy. It also carries out certain statistical explanations. The five BRICS countries were established for their own economic construction to be more stable in the international community, focusing on economic development and taking into account other development contents. The problem of severe natural disasters in today's world is increasing in frequency in both developed and developing countries [16]. Environmental problems and the emerging climate change have threatened the survival of human beings to a certain extent, and the corresponding legal measures adopted by various countries have also been gradually implemented in the form of articles. Since the content of the BRICS economic development is industry and manufacturing, it is necessary to compare the differences in environmental protection among the five countries. The differences in the environmental protection scores of the BRICS countries in the 2018–2019 years are presented in Table 1.

The data in Table 1 are the scores of the BRICS countries on different indicators of environmental protection, and this scoring system is based on the scoring results of different indicators of environmental protection in the five countries. Taking into account the comprehensiveness of the evaluation of the BRICS countries, the evaluation indicators of this Office are the natural resources possessed by the country, the integrity of environmental resources, the maximum bearing capacity of the natural environment, the management ability of environmental resources, and the ability to coordinate and allocate resources. In 2018–2020, the ratings of all BRICS countries improved, except for Russia, which declined. Among them, the improvement of China's score is the most obvious, and the improvement of the ranking has reached 24. The second obvious improvement is India, followed by Brazil and South Africa. It can be seen from Table 1 that the measures for environmental protection in the BRICS countries have achieved a more obvious effect on the sustainable impact of the environment [17]. In addition to scoring the environmental protection of each of the five countries above, in order to realize the implementation of the environmental protection law while taking into account economic development, that is, the corresponding national income brought by environmental protection, it needs to count the country's gross national product and the income brought by environmental protection. The results are shown in Table 2.

Table 2 compares Russia as GDP and environmental protection income. As a result, it can be seen that with the gradual increase of Russia's GDP in successive years, the income brought by environmental protection has also gradually increased. It can be seen that although the investment in environmental protection is low in short-term income, the overall income in the future is still very promising, because the generation of environmental protection income also means the implementation of environmental protection laws, including related legal taxes [18]. It is selected according to the indicators in Figure 2, and also statistics on the pollutants of sewage, gas, and waste residues produced by Russia's industries in the BRICS countries in different years. The results are shown in Table 3.

In Table 3, the corresponding statistics of the three types of pollutants in Russia in the past 10 years are carried out. The statistical results of these pollutants can clearly see that the total amount is increasing year by year. However, in the past three years, that is, 2018–2020, the discharge of pollutants has shown a decreasing trend. This is closely related to the enhancement of environmental protection by the BRICS countries in recent years. The above statistical content adopts the empirical analysis method and uses the relevant formula to deal with it.

Impact of BRICS Environmental Protection Laws on Economic Development: The five BRICS countries all play an important role in the development of today's world. Although they are all developing countries, the development potential contained in these five countries is huge. When developed countries transfer their own industries to developing countries, it brings economic development to developing countries and also brings environmental damage to developing countries. Although the BRICS countries have promulgated relevant environmental laws many years ago, the effect of implementation is not significant. In recent years, both the international community and the BRICS countries have paid more and more attention to the frequent occurrence of natural disasters. The tax system related to environmental law has also been improved accordingly, and this system has a great effect on the implementation of laws related to environmental protection [19]. Now, the relevant taxes and their proportions of environmental protection in Brazil and Russia in the past 10 years are counted, and the results are shown in Figure 5.

As can be seen from Figure 5, Brazil and Russia in the BRICS countries are increasing their investment in the environment year by year. This reflects the determination of the BRICS countries for environmental protection, and at the same time, it also reflects the good state of their own economic development. The laws of Brazil and Russia's investment in the environment are consistent, and the total investment in 2015 and before has gradually increased. Brazil's investment is 21.71 billion yuan, and Russia's investment is stable after 42.38 billion yuan. Correspondingly, the environmental protection tax has been increasing year by year, and the growth rate in Brazil and Russia from 2016 to 2020 reached 1.49% and 13.59%, respectively. Among them, Russia has the largest increase in returns on poster tax [20]. The above content calculates the attributes of economic development and environmental protection in the BRICS countries through formula (3).

Results of Environmental Sustainability Impacts: For environmental protection, developing countries will not take economic development as compensation. Although the development of industries has brought great damage to the environment, industry is very important to the economic development of a developing country. Since the industry needs to use a lot of energy in the process of development, in order to deal with the environmental pollution caused by traditional energy, this article will carry out quantitative empirical analysis of traditional energy and renewable energy. The result is shown in Figure 6.

The results in Figure 6 show the shift in energy usage. Traditional industrial energy is habitually used in most cases due to its high utility and adaptability, and the use of this energy is also increasing year by year [21]. It can be seen from the figure that due to the increase in the speed of development of the BRICS countries, the use of energy in the world's energy use continues to increase. By 2020, the BRICS countries will use 41.17% of industrial energy. But its use of renewable energy increased by 2.22% in 4 years 2017–2020, which reached 34.01%. Although it is not as good as the use of traditional energy, this result shows the efforts made by the BRICS countries for environmental protection. In order to better describe the attribute relationship between environmental protection and renewable energy, it needs to be calculated and defined using formula (1) and formula (3). In addition to the content discussed above, it also requires some specific and quantitative pollutant indicators for the BRICS countries in the implementation of environmental protection laws. It uses formula (6) to sum up the emissions of various pollutants, and the result is shown in Figure 7.

Figure 7 compares the emissions of pollutants in four BRICS countries. The results show that Russia and India are constantly increasing their pollutant emissions. By 2020, Russia's total emissions of polluting gases will reach 1,257 million tons, and India's total emissions of polluting gases will reach 2,271 million tons in the same year. This result shows that among the selected countries, countries with a faster development rate will produce more polluting gases. Together with the solution of the weight of formula (4), it can be known that the proportion of pollution caused by gas pollutants reaches 35.1%. After the environmental protection law was implemented in the form of taxation, the proportion of this pollutant dropped to 21.1%. It shows that the promulgation and implementation of environmental protection laws have a positive impact on the environment of the BRICS countries [22, 23].

## 3. Conclusion

This article is a discussion of environmental protection in the emerging economies of the BRICS in developing countries. This group of five developing countries has made its own contribution to global development in many ways. As typical representatives of developing countries, the BRICS countries have always been committed to the development of their own economic strength and comprehensive strength. Against the background of the common pursuit of environmental protection in today's international community, the BRICS countries are also carrying out environmental protection through some of their own actions. Compared with developed countries, the BRICS countries started a little late in protecting the environment due to their own development needs. In addition, the country's needs for industry and manufacturing make it difficult to coordinate the protection and destruction of the environment. At this stage, in order to implement the environmental law and better evaluate the effect of the environmental protection law, this article conducts an empirical analysis on environmental and economic development, as well as pollutants in the environment. It makes the article's elaboration on the sustainable impact of environmental protection law on the environment more complete.

## Figures and Tables

**Figure 1:** New model of environmental protection and economic development.

**Figure 2:** Evaluation system of the national secondary industry.

**Figure 3:** Secondary industry pollutant indicator system.

**Figure 4:** Sustainable development model under environmental protection.

**Figure 5:** Comparison of results of environmental investment and environmental taxation in Brazil and Russia. (a) Statistical results of environmental taxation and environmental investment in Brazil. (b) Statistical results of Russian environmental taxation and environmental investment.

**Figure 6:** Share of BRICS countries in world energy over 8 years.

**Figure 7:** Pollutant gas emissions of the 4 BRICS countries.

**Table 1:** Comparison of BRICS environmental protection scores in 2018–2020.

Nation	2018		2020		2018–2020 differences	
	Evaluation results	Score ranking	Evaluation results	Score ranking	Evaluation results	Score ranking
China	49.30	45	51.30	21	2.00	24
Russia	48.60	78	48.30	80	−0.03	−2
India	47.20	83	48.70	75	1.50	8
Brazil	52.10	21	52.70	17	0.60	4
South Africa	47.90	82	48.50	79	0.50	3

**Table 2:** Statistics of Russia's gross national product and environmental protection income.

years	Gross national product	Environmental protection income
2013	22940 billion	113.7 billion
2014	20820 billion	317.3 billion
2015	13700 billion	327.5 billion
2016	12800 billion	653.7 billion
2017	15740 billion	753.3 billion
2018	16610 billion	987.3 billion
2019	16880 billion	1013.7 billion
2020	14870 billion	1223.1 billion

**Table 3:** Generation of pollutants.

years	Sewage production	Harmful gas generation	Waste residue generation
2011	137.5 billion tons	127.3 billion tons	141.7 billion tons
2012	137.9 billion tons	138.7 billion tons	153.7 billion tons
2013	138.1 billion tons	152.6 billion tons	163.1 billion tons
2014	138.7 billion tons	153.8 billion tons	167.1 billion tons
2015	139.3 billion tons	154.6 billion tons	168.3 billion tons
2016	139.7 billion tons	157.5 billion tons	183.7 billion tons
2017	151.1 billion tons	158.9 billion tons	191.7 billion tons
2018	152.9 billion tons	161.7 billion tons	195.3 billion tons
2019	152.7 billion tons	160.7 billion tons	194.1 billion tons
2020	152.5 billion tons	159.3 billion tons	193.5 billion tons

## Data Availability

The data used to support the findings of this study are available from the corresponding author upon request.
